# A disintegrin and metalloprotease 17 promotes microglial cell survival via epidermal growth factor receptor signalling following spinal cord injury

**DOI:** 10.3892/mmr.2015.3395

**Published:** 2015-02-27

**Authors:** ZIJIAN WEI, DESHUI YU, YUNLONG BI, YANG CAO

**Affiliations:** 1 Graduate School of Liaoning Medical University, Jinzhou, Liaoning 121001, P.R. China; 2 Department of Orthopedics, The First Affiliated Hospital of Liaoning Medical University, Jinzhou, Liaoning 121001, P.R. China

**Keywords:** a disintegrin and metalloprotease 17, microglial cell survival, spinal cord injury, epidermal growth factor receptor signalling

## Abstract

Tumour necrosis factor-α (TNF-α) converting enzyme (TACE), also termed a disintegrin and metallopro-tease 17 (ADAM17), is involved in multiple cell signalling pathways. Through the secretion of epidermal growth factor receptor (EGFR) ligands, ADAM17 can activate the EGFR and is involved in various downstream signalling pathways. The present study aimed to investigate whether ADAM17-induced EGFR transactivation is involved in microglial cell survival following spinal cord injury (SCI). Reverse transcription quantitative polymerase chain reaction and western blot analysis revealed that ADAM17 was overexpressed in a mouse model following SCI. A 3-(4,5-dimethylthiazol-2-yl)-2,5-diphenyltetrazolium bromide assay demonstrated that the viability of human microglia and oligodendrocytes were significantly reduced in a time- and dose-dependent manner following treatment with the ADAM17 antagonist, TNF protease inhibitor 2. Hoechst 33258 staining and flow cytometric analysis revealed that inhibiting ADAM17 increased the rate of cellular apoptosis in neuronal and glial cell cultures, which was accompanied by increased cleavage of caspase-3. Western blot analysis demonstrated that inhibiting ADAM17 resulted in a reduction in the phosphorylation of the EGFR signalling pathway components and thereby impaired functional recovery, inhibited cell viability and prompted microglial apoptosis following SCI. Pre-treatment with the EGFR inhibitor, AG1478, rescued the ADAM17-mediated proliferation of microglial cells. These data demonstrated that ADAM17 contributed to microglial cell survival, predominantly by EGFR signalling, following SCI.

## Introduction

A disintegrin and metalloprotease 17 (ADAM17) has been identified cell surface glycoprotein beloning to the disintegrin and metalloprotease families (1). As a sheddase, this enzyme sheds several membrane ligands resulting in their release and, thereby, regulating various biological functions (2). ADAM17 was originally observed to shed the membrane bound form of tumour necrosis factor α (TNF-α) and is, therefore, also termed a TNF-α-converting enzyme (TACE) (2). Previous investigation has demonstrated that ADAM17 activates a variety of epidermal growth factor receptor (EGFR) ligands by shearing, thereby promoting tumour cell proliferation, invasion and metastasis (3). ADAM17 can activate EGFRs through the bidirectional protein regulation to improve the proliferation and invasion of cells in head and neck squamous cell carcinoma (4). Oyinbo *et al* confirmed that, through its shedding mechanism, ADAM17 is involved in metastatic squamous cell carcinoma (5). In addition, ADAM17 can enhance the invasiveness of glioma cells in a hypoxic environment, which is associated with activation of the EGFR signalling pathway (6).

The major signalling pathways of the EGFR include the Ras-Raf-mitogen-activated protein kinase (MAPK) signalling pathway (7). There are three major MAPK members, including extracellular signal-regulated kinases (ERKs), c-Jun N-terminal kinases (JNKs) and p38. The Ras-Raf-MAPK pathway predominantly regulates cell survival, proliferation and differentiation by regulating the expression of various genes. ERK1 and 2 are two subtypes of MAPK (8) and changes in the expression and distribution of ERK1/2 in cells indicates alterations in the MAPK signalling pathway (9). ERKs are predominantly involved in the regulation of mitogen-activated proliferation/differentiation factors, including E-cadherin, matrix metalloprotease (MMP)-2 and MMP-9, whereas the JNK and p38 MAPKs are closely associated with apoptosis (10). The activation of JNK usually leads to the abnormal expression of proliferation associated proteins, including the B-cell lymphoma-extra large (BclxL) and X-linked inhibitor of apoptosis protein (XIAP) anti-apoptotic genes. By contrast, p38 MAPKs cause cell cycle arrest and apoptosis through a series of target genes, including p27^Kip1^, Bcl-2-interacting mediator of cell death, BclxL and XIAP (11).

Spinal cord injury (SCI) induces a marked post-traumatic inflammatory response, which causes secondary injury and results in limited functional recovery (12). Several studies have observed increased levels of pro-inflammatory cytokines, including TNF-α, within hours of injury (12,13). Therefore the increased expression of TNF-α is associated with cell apoptosis, increased vascular permeability and reduced glutamate metabolism (14,15). Pro-TNF-α exists as a type II transmembrane protein and is released by ADAM17 through the proteolytic cleavage of the membrane-bound form. When TNF-α is released, it exerts a marked inflammatory response in various organs. It has been suggested that mice lacking ADAM17 in lymphocytes, demonstrate antibacterial sepsis capabilities due to the cell being unable to shed the membrane-bound TNF-α (16). Therefore, ADAM17 inhibitors may observe efficacy in rheumatoid arthritis and multiple sclerosis models, since ADAM17 has been demonstrated to reduce the production of soluble TNF-α and decrease inflammation (17). However, the role of EGFR signalling on ADAM17-induced microglial cell survival following spinal cord injury remains to be elucidated.

The present study investigated the role of ADAM17 on microglial cell survival which may contribute to the treatment of SCI.

## Materials and methods

### Human cell lines

Human microglia and oligodendrocyte cell lines were purchased from American Type Tissue Culture Collection (Manassas, VA, USA) and cultured in Dulbecco’s modified Eagle’s medium (DMEM)/F12 (GE Healthcare, Logan, UT, USA) supplemented with 10% fetal bovine serum (FBS; GE Healthcare), 100 U/mL penicillin (Solarbio, Beijing, China) and 100 U/mL streptomycin (Solarbio) in a 25 cm^2^ culture flask (Corning, Inc., Corning, NY, USA) at 37°C in a humidified atmosphere with 5% CO_2_.

### Experimental animals

All animal procedures were performed in accordance with the National Institutes of Health Animal Care and Use Guidelines (1). All animal procedures were approved by the Animal Ethics Committee at the Liaoning Medical University (Jinzhou, China). A total of 12 10-week old C57BL/6 male mice were purchased from Vital River aboratory Animal Technology Co., Ltd. China (Beijing, China). Animals were fed a standard laboratory diet and recovered for two weeks at 24°C in a humidity controlled environment under a 12-h light/dark cycle.

### Isolation of primary neuronal cells

Spinal cord segments T8-T10 of non-injured or contusion spinal cord injured (injury at T9) mice were dissected and mechanically dissociated with fine scissors in Hank’s Balanced Salt Solution (HBSS; Hyclone, Logan, UT, USA) at room temperature. Prior to tissue dissociation, whole spinal cord columns were kept on dry ice for 5 min prior to the extraction of cord segments T8-T10. Tissue was retrieved by centrifugation (1 min, 400 × g, room temperature) and enzymatically dissociated with 2.5 mg trypsin and 5 mg collagenase (Sigma-Aldrich, St. Louis, MO, USA) in 5 ml DMEM for 20 min at 37°C. DMEM (10 ml) and 10% fetal bovine serum were added to the cells to inhibit enzymatic activities and then was filtered through a 40 *μ*m cell strainer. Dissociated spinal cells in HBSS (6 ml) were layered on top of the OptiPrep gradient (Sigma-Aldrich) before centrifugation (15 min, 400 × g, 20°C), separating the cell solution into distinct layers with debris on top, followed by three layers of neurons, and inflammatory cells, glia and red blood cells in the pellet. The debris layer was carefully aspirated. The remaining cells were cultured in mixed cultures for 2 days at 37°C. The medium was refreshed with high glucose DMEM containing 20% FBS. The microglial cells were isolated 10 days later using an orbital shaker (37°C, 200 rpm, 2 h; TS-200, Qilin-lab Industrial Inc., Haimen, China). At 30 min post-isolation, the medium was refreshed for further purification. The cells were then identified using a CD11b antibody and cultures with a purity of >97% identified via flow cytometry (FACSCalibur; BD Biosciences, Franklin Lakes, NJ, USA) were used for subsequent experiments.

### Transfection of microglia cells with ADAM17 cDNA

The cDNA encoding ADAM17 was purchased from OriGene Technologies, Inc. (Rockville, MD, USA) and the pcDNA3.1 control vector was purchased from Invitrogen Life Technologies (Carlsbad, CA, USA). Briefly, 2×10^6^ microglial cells were resuspended in a nucleofector reagent of a Cell Line Nucleofector kit V (Amaxa Biosystems, Gaithersburg, MD, USA) mixed with 2 *μ*g cDNA and pulsed, according to the manufacturer’s instructions. Immediately following nucleofection, 5000 cells/cm^2^ were transferred into six wells containing 200 *μ*l/cm^2^ (DMEM)/DF12 culture medium and incubated at 37°C for 48 h prior to selection using Geneticin (Invitrogen Life Technologies).

### Modified cell lines and inhibitors

The modified cell lines used were microglial cells stably transfected with the ADAM17 cDNA plasmid (OriGene) or with a vector control plasmid of pCMV6-XL4 (OriGene). The ADAM17 inhibitor, TAPI-2, was purchased from Peptides International, Inc. (Louisville, KY, USA) and the EGFR phosphorylation inhibitor, AG1478, was purchased from Sigma-Aldrich (St. Louis, MO, USA). AG1478 was reconstituted in freshly prepared phosphate-buffered saline (PBS; pH 3.5; Zhongshanjinqiao, Beijing, China). For the *in vitro* investigation, TAPI-2 was used at a concentration of 0.1, 1 or 3 mM and the *in vivo* experiments with TAPI-2 were performed using 2.2 mM (210 mg/day).

### Spinal cord T-cut hemisection injury

The T-cut hemisection injury was performed, as described previously (18). Briefly, the mice were anesthetised by intraperitoneal injection with 4% chloral hydrate (100 *μ*l/100 g body weight) and underwent a partial laminectomy at thoracic level T8. The mice were subjected to a bilateral dorsal T-cut hemisection using iridectomy scissors to transect the left and right dorsal funiculus, the dorsal horns and the ventral funiculus. This injury procedure causes complete transection of the dorsomedial and ventral corticospinal tract and induces the impairment of several other descending and ascending tracts (18). The muscles were sutured with 4–0/T mucosal sutures and the back skin was closed with wound clips (Solarbio). Sham-injured mice received a laminectomy without weight drop. Following surgery, the mice were placed in a temperature- (20–24°C) and humidity-controlled (45–55%) environment under a 12-h light/dark cycle until they were awake and then returned to their original cage. The bladders of the mice were manually voided daily until the mice were capable of urinating independently.

### Assay of cell viability

The cell viability was determined using a colorimetric, 3-(4,5-dimethylthiazol-2-yl)-2,5-diphenyltetrazolium bromide (MTT) assay (Sigma-Aldrich). To determine the impact of ADAM17 on cell viability, the microglia and oligodendrocytes were cultured at ~70% confluence and starved in serum-free DMEM overnight. The microglia and oligodendrocytes were pre-incubated with 0.1, 1 or 3 mM TAPI-2, the ADAM17 antagonist, at 37°C in serum-free DMEM for 48 h. Following treatment, the cells were cultured in fresh DMEM containing 0.5 mg/ml MTT for 4 h at 37°C. Dimethylsulfoxide was then added to the wells to dissolve the blue formazan products and the absorbance was measured spectrophotometrically at a wavelength of 550 nm (xMark; Bio-Rad Laboratories, Inc., Hercules, CA, USA). To determine the time-dependent effects, the cells were pre-incubated in DMEM at 37°C with 1 mM TAPI-2 for 12, 24 and 48 h and cell viability was determined, as described above. Each experiment was performed independently at least three times.

### Hoechst 33258 staining

The human microglia and oligodendrocytes (1×10^5^ cells/well) were cultured in 6-well tissue culture plates in DMEM with 10% FBS at 37°C. At 70–80% confluence, the cells were incubated for 16 h in serum-free DMEM and then 1 mM TAPI-2 was added to the fresh media for 48 h. Following drug treatment, the media was removed and the cells were rinsed three times with cold PBS and fixed using 4% formaldehyde (Zhongshan Gold Bridge Biological Technology Co., Beijing, China) in PBS for 20 min at room temperature. The cells were then washed three times with cold PBS and stained with Hoechst 33258 (10 *μ*g/ml; Sigma-Aldrich) for 5 min. Following staining, the cells were further washed with cold PBS and examined under a fluorescence microscope (DM IRB; Leica Microsystems GmbH, Wetzlar, Germany).

### Western blot analysis

Mouse spinal cord tissue (5 mm) centered around the injury site was obtained 1, 3, 7, 14 and 28 days after injury (n=4 mice per time-point) and four laminectomy-only mice were used as a control. The proteins were extracted using radioimmunoprecipitation buffer (Solarbio) containing 50 mM Tris/HCl (pH 7.4), 150 mM NaCl, 1% (v/v) NP-40 and 0.1% (w/v) sodium dodecyl sulphate (SDS) with 1% (v/v) phenylmethanesulfonylfluoride (Solarbio), 0.3% (v/v) P8340-1ML Protease Inhibitor Cocktail (Sigma-Aldrich) and 0.1% (v/v) phosphorylated proteinase inhibitor (Sigma-Aldrich). The supernatants were extracted from the lysates following centrifugation at 15,000 × g at 4°C for 15 min. To quantify the relative concentration of the total proteins, a Bicinchoninic Acid Protein Assay kit (Pierce Biotechnology, Inc., Rockford, IL, USA) was used. The proteins (15 *μ*g) were separated on an 10% SDS-PAGE gel and transferred onto a polyvinylidene fluoride (PVDF; Qiagen, Hilden, Germany) membrane at 300 mA for 2 h. To inhibit non-specific binding, the PVDF membrane was blocked using 8% (w/v) non-fat milk in Tris-buffered saline containing Tween-20 for 2 h at room temperature. The membranes were then incubated with primary antibodies against β-actin, phosphorylated (p-)EGFR (#3777; monoclonal rabbit IgG), EGFR (#4267; monoclonal rabbit IgG), p-ERK1/2 (#4370; monoclonal rabbit IgG), ERK1/2 (#9102; polyclonal rabbit), p-JNK (#81E11; monoclonal rabbit IgG), JNK (#2C6; monoclonal mouse IgG1), p-p38 (#D3F9; monoclonal rabbit IgG), p38 (#D13E1; monoclonal rabbit IgG), Bcl-2 (#50E3; monoclonal rabbit), Bax (#D2E11; monoclonal rabbit IgG) and caspase-3 (#8G10; monoclonal rabbit IgG) (1:1,000; Cell Signaling Technology, Inc., Danvers, MA, USA) overnight at 4°C. The membranes were washed with PBS containing 0.1% Tween-20 (PBST; Solarbio) four times (5 min each) prior to incubation with a horseradish peroxidase-conjugated goat anti-rabbit immunoglobulin G (1:5,000; Abmart, Shanghai, China) for 2 h at room temperature. Following antibody incubation, the membranes were washed, as previously, followed by Fusion SL 3500 enhanced chemiluminescence detection (Merck Millipore, Darmstadt, Germany) was performed, according to the manufacturer’s instructions. The relative protein level was determined and changes in the protein expression of the target protein was normalised relative to β-actin.

### Apoptosis assay

To determine the effects of ADAM17 on microglia and oligodendrocyte apoptosis, the cells (50–60% confluent) were treated with 0.1, 1 or 3 mM TAPI-2, the ADAM17 antagonist, for 48 h at 37°C. Following treatment, the cells were washed three times with 1X PBS. An Annexin V-Fluorescein isothiocyanate (FITC)-Propidium Iodide (PI) Apoptosis kit (Invitrogen Life Technologies) was used to determine the apoptotic rate by flow cytometry. This assay uses fluorescein-labelled annexin V with PI to detect cells undergoing apoptosis. Briefly, the cells were washed with 1X PBS three times and 2–3×10^6^ cells/ml were incubated in 1X annexin V binding buffer (200 *μ*l) containing 10 mM HEPES/NaOH (pH 7.4), 140 mM NaCl and 2.5 mM CaCl_2_ at room temperature for 15 min in the dark. The annexin V-FITC and PI buffer were added to the cells and incubated at room temperature for 15 min in the dark. Untreated cells were used as internal control. Following incubation, the cells were filtered using a filter screen (Zhongshanjinqiao) and analysed by flow cytometry (EPICS^®^ ALTRA™; BD Biosciences) within 1 h of staining, using FITC and PI lasers.

### Statistical analysis

The data are expressed as the mean ± standard error of the mean. The number of independent experiments is represented by ‘n’. Multiple comparisons were performed using a one-way analysis of variance followed by Tukey’s multiple-comparison test. P<0.05 was considered to indicate a statistically significant difference. GraphPad Prism 5 (GraphPad Software, Inc., La Jolla, CA, USA) was used for all statistical analyses.

## Results

### Upregulation of ADAM17 following SCI

To evaluate the effect of SCI on the protein levels, changes in the expression of ADAM17 were determined between 1 and 28 days following SCI. Quantitative analysis of western blotting revealed that the expression of ADAM17 was rapidly increased following SCI (Fig. 1A and B).

### Microglia and oligodendrocyte cell viability is affected by an ADAM17 antagonist in a dose- and time-dependent manner

To investigate the effect of ADAM17 on cell viability, human microglia and oligodendrocytes were treated with 0.1, 1 or 3 mM of the ADAM17 antagonist, TAPI-2, for 48 h. Cell viability was assessed using an MTT assay. As shown in Fig. 2A, the cell viability of human microglia and oligodendrocytes was significantly reduced by ~30% when the concentration of TAPI-2 was increased between 0 and 3 mM. Furthermore, human microglia and oligodendrocytes were treated with 1 mM TAPI-2 for 12, 24 and 48 h, and the corresponding cell viability was determined using an MTT assay. The viability of the human microglia and oligodendrocytes was reduced by ~11 and 16% at 24 and 48 h, respectively (Fig. 2B). This suggested that the viabilities of human microglia and oligodendrocytes were significantly reduced by TAPI-2 in a dose- and time-dependent manner.

### Inhibition of ADAM17 increases the apoptosis of microglia and oligodendrocytes in vitro

Human microglia and oligodendrocytes were treated with 1 mM TAPI-2 for 48 h and the cells were stained with Hoechst 33258. As shown in Fig. 3A, increased cell apoptosis was observed following incubation of the cells with TAPI-2. To quantify the percentage of apoptotic cells, an annexin V-PI kit was used. Flow cytometry revealed that treatment with 1 mM TAPI-2 increased the number of apoptotic cells by 87, 100 and 132 % compared with the control (Fig. 3B). To further examine the effects of ADAM17 on human microglia and oligodendrocyte apoptosis, alterations in the expression levels of apoptosis-associated proteins were assessed by western blot analysis. Following treatment of the human microglia and oligodendrocytes with 1 mM TAPI-2 for 48 h, the expression of cleaved caspase-3 increased (Fig. 3C and D). Caspase-3 is present as an inactive zymogen within the body, however, during apoptosis, caspase-3 is hydrolysed and becomes an active enzyme (19). Following the increased expression of cleaved caspase-3, the expression of Bax increased and the expression of Bcl-2 decreased. These results suggested that TAPI-2 induced the apoptosis of human microglia and oligodendrocytes predominantly by increasing the expression of cleaved caspase-3.

### Overexpression of ADAM17 confers cell survival in microglia and oligodendrocytes

To determine the biological relevance of the upregulation of ADAM17, microglia and oligodendrocytes overexpressing ADAM17 were generated. Western blot analysis of the apoptosis effector molecules revealed that overexpression of ADAM17 significantly (P<0.01) reduced the expression levels of cleaved caspase-3 and Bax, compared with the empty vector control cells (Fig. 4A and B).

### ADAM17-mediated cell survival involves activation of the EGFR/MAPK signalling pathway

The present study investigated whether the EGFR/MAPK signalling pathway was involved in cell survival, conferred by inhibiting ADAM17. As shown in Fig. 5A, downregulation of ADAM17 in mice following SCI caused a significant reduction in the expression levels of p-EGFR, p-JNK, p-ERK1/2 and p-p38, compared with the control mice. However, the total protein levels of EGFR, JNK, ERK1/2 and p38 remained stable. Flow cytometric analysis demonstrated that pre-incubation with the EGFR inhibitor, AG1478, reversed the effects of overexpression of ADAM17 and increased cell survival (Fig. 5B). These results indicated that the ADAM17-mediated survival of microglia and oligodendrocytes involved activation of the EGFR/MAPK signalling pathway.

## Discussion

ADAM17 is involved in various cell signalling pathways and, as a sheddase, has important functions in cell survival and apoptosis (4). The present study investigated the specific function of ADAM17 in microglia survival following SCI. The specific ADAM17 inhibitor, TAPI-2, and an ADAM17-overexpression vector were used to demonstrate that ADAM17 promoted the survival of microglia *in vitro* and *in vivo*.

In glioma cells, ADAM17 increases the invasiveness of brain tumour proteolytic activity under hypoxic conditions (20). In addition, the tumour growth and tissue invasion capacities are significantly reduced following ADAM17-knockdown in human renal carcinoma cells (21,22). The EGFR signalling pathway is important for cell survival and ADAM17 has been identified as the predominant sheddase for a number of EGFR pro-ligands (23,24). The EGFR ligand-banding leads to the receptor self-dimerisation, autophosphorylation and subsequent activation of the downstream Ras/MAPK/ERK signalling pathways (3). EGFR belongs to the family of tyrosine kinases involved in cell differentiation, proliferation and survival. Following binding of EGFR with the ligands, it combines with the other EGFR monomers thereby exerting downstream effects (25).

The present study aimed to examine the activation of the EGFR signalling pathway by ADAM17 in microglia and oligodendrocytes. The *in vivo* data indicated that ADAM17 was significantly increased following SCI. The inhibition of ADAM17 by TAPI-2 significantly inhibited cell viability in a dose- and time-dependent manner (Fig. 2A and B). Furthermore, the cell apoptotic rates were significantly increased following pre-incubation of microglia and oligodendrocytes with 1 mM TAPI-2 for 48 h. When ADAM17 was inhibited by TAPI-2, the expression of activated caspase-3 significantly increased, therefore, microglia and oligodendrocytes were more susceptible to cell apoptosis and death. By contrast, the stable transfection of microglia with a vector overexpressing ADAM17 or an empty vector revealed significant effects on cell survival, which enabled the functional recovery of microglial cells following SCI.

ADAM17 regulates the domain shedding of various pro-ligands, therefore, the present study investigated the EGFT signalling pathway, an important cellular pathway associated with cell survival and ADAM17 (2,3). Mice, which were fed with the ADAM17 antagonist, TAPI-2, had a reduced expression of p-EGFR, demonstrating that the inhibition of EGFR reduces the MAPK/JNK/ERK signalling cascade by modulating the apoptotic response following SCI. Inhibition of EGFR signalling reduced the survival of microglia and oligodendrocytes and the functional recovery of mice following SCI. Previous studies have demonstrated that microglia activation positively correlates with the activation of EGFR, indicating that EGFR may be a potential therapeutic target for SCI (26). *In vitro* and *in vivo* investigations have revealed that EGFR is significantly phosphorylated in activated microglia and that inhibition of EGFR results in reduced activation of microglia. The present study revealed that the inhibition of the phosphorylation of EGFR results in an increased microglial apoptotic response. By contrast, overexpression of ADAM17 reduced the rate of apoptosis, observed by flow cytometry. The inhibition of EGFR did not reduce the apoptotic response when ADAM17 was overexpressed (Fig. 5B). These results indicated that ADAM17 promoted microglial cell survival predominantly by activating the EGFR signalling pathway.

The present study demonstrated that the inhibition of ADAM17 reduced the phosphorylation of EGFR in human microglia and oligodendrocytes and in mice. However, the underlying mechanism remains to be elucidated. A previous study reported MAPK, JNK and ERK1/2 as three primary downstream pathways of the EGFR cascade (27). MAPKs are important for regulating cellular proliferation, inflammatory responses and other biological activities (28). The present study indicated that the EGFR signalling pathway was activated by ADAM17. These results suggested that the overexpression of ADAM17 promoted microglial cell survival following SCI, predominantly through regulating the activation of the EGFR/MAPK/JNK/ERK1/2 cascade. EGFR signalling is considered to be neuroprotective and it is now a recognised therapeutic target (29). EGFR protects the brain from injury, exerting a neuroprotective function (30). Furthermore, EGFR induces cell survival following central nervous system (CNS) disorders (31), with rapid activation of the EGFR signalling pathway following CNS disorders, including stroke and Alzheimer’s disease (32). Therefore, the specific mechanism underlying the association between ADAM17 and EGFR following SCI requires further investigation.

## Figures and Tables

**Figure 1:** Expression of ADAM17 in spinal cord tissue samples from 1–28 days following spinal cord injury. (A) Representative western blot and (B) the expression ratio of ADAM17 to GAPDH are presented. The data are expressed as the mean ± standard deviation. Statistical analysis was performed using a one-way analysis of variance followed by Tukey’s test (n=3; ^**^P<0.01, vs. 0 day control group). ADAM17, A disintegrin and metalloprotease 17.

**Figure 2:** Human microglial and oligodendrocyte cell viability is affected by TAPI-2 in a dose- and time-dependent manner. (A) Human microglia and oligodendrocytes were exposed to TAPI-2 (0.1, 1 or 3 mM) for 48 h. (B) Human microglia and oligodendrocytes were treated with 1 mM TAPI-2 for 12, 24, and 48 h. Cell viability was determined using an MTT assay at 550 nm. Data are expressed as the mean ± standard deviation (n=6; ^*^P<0.05, vs. control). OD, optical density.

**Figure 3:** Human microglial and oligodendrocyte apoptosis increased following incubation of the cells with 1 mM TAPI-2 for 48 h. (A) Hoechst 33258 staining demonstrated increased apoptosis (magnification, ×40). (B) An annexin V-PI kit was used to detect cell apoptosis. Caspase-3 was activated when (C) human microglia and (D) oligodendrocytes were treated with 1 mM TAPI-2 for 48 h. The data are expressed as the mean ± standard deviation (n=3; ^*^P<0.0 and ^**^P<0.01, vs. Con). Con, control, ADAM17, A disintegrin and metalloprotease 17; Bcl-2, B cell lymphoma; Bax, Bcl-2 associated X protein, DAPI, 4′6-diamidino-2-phenylindole; TAPI-2, TNF protease inhibitor 2; PI, propidium iodide.

**Figure 4:** Overexpression of ADAM17 attenuates apoptosis in microglia and oligodendrocyte cells. Western blot analysis was performed to measure the expression levels of ADAM17 and apoptosis effector molecules, cleaved caspase 3, Bcl-2 and Bax, in (A) microglia and (B) oligodendrocytes transfected with pADAM17 or the pcDNA3.1 empty vector control. The data are expressed as the mean ± standard deviation (n=3; ^*^P<0.05 and ^**^P<0.01, vs. control). ADAM17, A disintegrin and metalloprotease 17; Bcl-2, B cell lymphoma; Bax, Bcl-2 associated X protein; p, plasmid.

**Figure 5:** Involvement of the EGFR/MAPK signaling pathway in ADAM17-mediated cell survival. (A) Western blot analysis was performed to measure the expression levels of p-EGFR and p-MAPK in mice fed 2.2 mM TAPI-2 per day. (B) Flow cytometry bar graphs show the apoptotic ratio in microglial cells transfected with either an ADAM17-overexpressing vector, an empty vector or pre-incubated and treated with the EGFRi. The data are expressed as the mean ± standard deviation (n=3; ^*^P<0.05 and ^**^P<0.01, vs. Con; ^#^P<0.05, vs. ADAM17+EGFRi. EGFR, epidermal growth factor receptor; MAPK, mitogen activated protein kinase; ADAM17, A disintegrein and metalloprotease 17; p-, phosphorylated; EGFRi, EGFR phosphorylation inhibitor (AG1478); Con, control; ERK, extracellular signal-regulated kinase; JNK, c-Jun N-terminal kinase; TAPI-2, TNF protease inhibitor 2.
